This article has been retracted.

# Transdermal Delivery of Insulin by Amidated Pectin Hydrogel Matrix Patch in Streptozotocin-Induced Diabetic Rats: Effects on Some Selected Metabolic Parameters

**DOI:** 10.1371/journal.pone.0101461

**Published:** 2014-07-02

**Authors:** Silindile I. Hadebe, Phikelelani S. Ngubane, Metse R. Serumula, Cephas T. Musabayane

**Affiliations:** Schools of Laboratory Medicine and Medical Sciences, University of KwaZulu-Natal, Durban, South Africa; Virgen Macarena University Hospital, School of Medicine, University of Seville, Spain

## Abstract

**Purpose:**

Studies in our laboratory are concerned with developing optional insulin delivery routes based on amidated pectin hydrogel matrix gel. We therefore investigated whether the application of pectin insulin (PI)-containing dermal patches of different insulin concentrations sustain controlled release of insulin into the bloodstream of streptozotocin (STZ)-induced diabetic rats with concomitant alleviation of diabetic symptoms in target tissues, most importantly, muscle and liver.

**Methods:**

Oral glucose test (OGT) responses to PI dermal matrix patches (2.47, 3.99, 9.57, 16.80 µg/kg) prepared by dissolving pectin/insulin in deionised water and solidified with CaCl_2_ were monitored in diabetic rats given a glucose load after an 18-h fast. Short-term (5 weeks) metabolic effects were assessed in animals treated thrice daily with PI patches 8 hours apart. Animals treated with drug-free pectin and insulin (175 µg/kg, sc) acted as untreated and treated positive controls, respectively. Blood, muscle and liver samples were collected for measurements of selected biochemical parameters.

**Results:**

After 5 weeks, untreated diabetic rats exhibited hyperglycaemia and depleted hepatic and muscle glycogen concentrations. Compared to untreated STZ-induced diabetic animals, OGT responses of diabetic rats transdermally applied PI patches exhibited lower blood glucose levels whilst short-term treatments restored hepatic and muscle glycogen concentrations. Plasma insulin concentrations of untreated diabetic rats were low compared with control non-diabetic rats. All PI treatments elevated plasma insulin concentrations of diabetic rats although the levels induced by high doses (9.57 and 16.80 µg/kg) were greater than those caused by low doses (2.47 and 3.99 µg/kg) but comparable to those in sc insulin treated animals.

**Conclusions:**

The data suggest that the PI hydrogel matrix patch can deliver physiologically relevant amounts of pharmacologically active insulin.

**Novelty of the Work:**

A new method to administer insulin into the bloodstream via a skin patch which could have potential future applications in diabetes management is reported.

## Introduction

The tight glycaemic control required to attenuate chronic complications in type 1 diabetes mellitus often requires numerous daily injections of bolus insulin [1] administered by subcutaneous (sc) needle injection, insulin pen and catheters connected to insulin pumps [2], [3]. These methods are, however, inconvenient and often lead to poor compliance, a major factor negating the quality of life of diabetic patients [4]–[8]. In addition, studies suggest that bolus insulin injections cause adverse effects such as hyperinsulinaemia, insulin resistance, glucose intolerance, weight gain and cardiovascular complications [9]–[13]. The key to strict glycaemic control with use of exogenous insulin lies in the creation of delivery methods that mimic the physiology of insulin secretion. The desire to deliver insulin conveniently and effectively has led to investigations of delivery systems such as oral, nasal, buccal, pulmonary, rectal, ocular and transdermal routes [14]–[16]. The skin which has increasingly become a route of the delivery for a wide range of drugs has generated a great deal of interest [17]. The route is an appealing alternative for insulin as this may offer patient compliance and controlled release over time by avoiding degradation in the gastrointestinal tract or first-pass liver effects [18]–[20]. On the other hand, transdermal delivery is limited by the low permeability of skin caused mainly by stratum corneum, the skin’s outermost layer [21]. However, the permeability can be increased by various techniques such as the use of chemical enhancers, electrical enhancers via iontophoresis or electroporation and ultrasonic enhancers [22]–[24].

Reports suggest that pectin (polygalacturonic acid) not only delivers drugs to the colonic region of the gastrointestinal tract, but also sustains drug release *in vitro* [25]. More interestingly, Musabayane et al., succeeded in sustaining plasma insulin concentrations in diabetic rats using orally administered, insulin-loaded amidated pectin hydrogel beads [14]. Building off these previous studies, we sought to develop a pectin insulin-containing dermal patch formulation which can transport insulin across the skin and sustain controlled release into the bloodstream of streptozotocin (STZ)-induced diabetic rats. The study was, therefore, designed to establish whether application of pectin insulin-containing dermal patches sustain controlled release of insulin into the bloodstream of STZ-induced diabetic rats with concomitant alleviation of some diabetic symptoms. The success of insulin delivery via this route can be assessed by the ability to lower blood glucose concentrations. In addition to reduced insulin responsiveness in muscle in diabetes, recent evidence has emphasized the critical role of insulin in hepatic glucose homeostasis [26]. Insulin exerts metabolic and cellular effects mediated through the insulin receptor (IR) that is present in virtually all vertebrate tissues including the skin [27]. Accordingly, the effects of insulin-containing dermal patches on the expression of insulin-stimulated enzymes and facilitative glucose transporters in insulin responsiveness target tissues, most importantly, muscle and liver of STZ-induced diabetic rats were also assessed.

## Materials and Methods

### Drugs and chemicals

Amidated low-methoxyl pectin with a degree of methoxylation (DM) of 23, degree of amidation (DE) of 24 was kindly donated by Dr Hans-Ulrich Endress of Herbstreith and Fox KG, Neuenburg, Germany. Drugs were sourced from standard pharmaceutical suppliers. All other chemicals which were of analytical grade quality were purchased from standard commercial suppliers.

### Patch preparation

Amidated pectin hydrogel insulin (PI) matrix patches of different insulin concentrations were prepared using a previously described protocol by Musabayane et al. [28] with slight modifications. Briefly, amidated low methoxyl pectin was dissolved in deionized water (4 g/100 mL) and mixed with agitation for 30 min. Subsequently, DMSO (3 mL, Sigma-Aldrich Chemical Company, Missouri, St Louis, USA), eucalyptus oil (1.5 mL, Barrs Pharmaceutical Industries cc, Cape Town, South Africa), vitamin E (1.5 mL, Pharma Natura Pty Ltd, Johannesburg, South Africa) and purmycin (100 µL, Pharmacare Ltd, Johannesburg, South Africa) were added to the mixture and left to spin for another 30 min after which various amounts of insulin (NovoRapid Pen Refill, Novo Nordisk Pty Ltd, Sandton, South Africa) were added to separate beakers and mixed with agitation in a water bath at 37°C for 15 min. Following this, aliquots (11 mL) were transferred to petri dishes with known diameter and 2% CaCl_2_ solution was added on top and left at room temperature for 10 minutes to allow for cross-linking and formation of the matrix patch. Preliminary studies indicated that the patches contained 0.74, 1.20, 2.87 and 5.04 µg of insulin which translated to dosages of 2.47, 3.99, 9.57 and 16.80 µg/kg, respectively.

### Determination of insulin amounts in patches

The pectin hydrogel matrix dermal patches of the same size were dissolved in Sorenson’s phosphate buffer (pH 7.2) to determine the amount of insulin incorporated. To assess the stability in the pectin hydrogel matrix formulation, the recovery percentages of insulin with the original insulin were monitored over a period of two months.

### Animals

Male Sprague-Dawley rats (250–300 g) bred at the Biomedical Research Unit, University of KwaZulu-Natal were used in this study. The animals were kept and maintained under standard laboratory conditions of temperature, humidity, 12 h day: 12 h night cycle, and allowed water *ad libitum* and given 30 g standard rat chow daily (Meadow Feeds, Pietermaritzburg, South Africa). All animal experimentation was reviewed and approved by the Animal Ethics Committee of the University of KwaZulu-Natal (102/11/Animal).

### Diabetic animal model

To generate type 1 diabetes mellitus animal model, male Sprague-Dawley rats were injected with single intraperitoneal injection of 60 mg/kg STZ (Sigma-Aldrich Chemical Company, Missouri, St Louis, USA) in freshly prepared 0.1 M citrate buffer (pH 6.3). The control group received the vehicle citrate buffer through the same route. Animals that exhibited glucosuria after 24 h, tested by urine strips (Rapidmed Diagnostics, Sandton, South Africa) were considered diabetic. Seven days later, the blood glucose concentration of STZ-induced diabetic rats greater than 20 mmol/L was considered as stable diabetes.

### Application of the hydrogel patch

Rats were shaved on the dorsal region of neck 1–2 days prior to the application of PI hydrogel matrix patches. The dermal patches were secured in place with adhesive hydrofilm (Hartman-Congo Inc, Rock Hill, South Carolina, USA) and rat jackets (Braintree, Scientific, Inc, Braintree, Massachusetts, USA) which were adjusted for the size of the animal.

### Blood glucose effects

OGT responses to application of PI-containing dermal patches of different insulin concentrations (2.47, 3.99, 9.57 and 16.80 µg/kg) were evaluated in separate groups of STZ-induced diabetic rats according to the method described previously by Musabayane et al. [29] with slight modifications. Briefly, separate groups of STZ-induced diabetic rats were fasted overnight (18 h), followed by monitoring of OGT responses to dermal matrix patches. Rats sham applied with drug free pectin dermal hydrogel matrix patches and insulin (175 µg/kg, sc) served as control animals and positive control animals, respectively. Blood glucose was measured using a glucometer (OneTouch select glucometer, Lifescan, Mosta, Malta, United Kingdom) at 15 min intervals for the first hour and then hourly for the subsequent 5 hours after glucose-loading (0.86 mg/kg). Matrix patches of different insulin doses (3.99, 9.57, 16.80 µg/kg) were topically applied onto the shaved skin area on the back of the neck skin three times a day 8 h apart (09h00, 17h00 and 01h00). Animals treated with drug-free pectin and insulin (175 µg/kg, sc) acted as negative and positive controls, respectively. Blood glucose concentration was measured daily at 09h00 using a glucometer (OneTouch select glucometer, Lifescan, Mosta, Malta, United Kingdom) whilst body weights, amounts of water and food consumed were recorded every 3^rd^ day.

### Pharmacokinetic studies

Blood samples were collected by cardiac puncture into pre-cooled heparinized tubes after 6 h from separate parallel groups of STZ-induced diabetic rats prepared as for OGT responses for insulin determination. Samples were also collected from all groups of animals by cardiac puncture into individual pre-cooled heparinized containers at the end of the 5-week experimental treatment period for insulin and biochemical measurements. The plasma insulin concentrations were measured by ultrasensitive rat insulin ELISA kit (DRG Instruments GmBH, Marburg, Germany). This immunoassay is a quantitative method utilizing two monoclonal antibodies which together are specific for insulin. The lower limit of detection was 1.74 pmol/L. The intra- and inter-assay analytical coefficients of variation ranged from 4.4 to 5.5% and from 4.7 to 8.9%, respectively.

### Tissue sample harvesting

All animals were sacrificed by exposing to halothane for 3 min via a gas anaesthetic chamber (100 mg/kg) at the end of the 5 week experimental period. Thereafter, skin samples and subcutaneous tissues around the dorsal region of neck where the patches were applied and insulin injection sites, as well as liver and gastrocnemius muscle tissues were removed, snap frozen in liquid nitrogen and stored in a BioUltra freezer (Snijers Scientific, Tilburg, Netherlands) at −70°C until use. All organs were analyzed for protein content in addition to other biochemical parameters.

### Glycogen measurements

The glycogen concentration was determined as previously described by Khathi *et al.* [30]. Liver and muscle tissue samples (1–1.5 g) were homogenized in 2 mL of 30% KOH solution and digested at 100°C for 30 min and then cooled in ice-saturated sodium sulphate. The glycogen was precipitated with ethanol and then pelleted, washed, and dissolved in deionized water. Glycogen standards (10–2000 mg/L) were also prepared using glycogen powder. The glycogen concentration was determined by its reaction with the anthrone reagent (2 g anthrone/1 of 95% (v/v) H_2_SO_4_) after which absorbance was measured at 620 nm using a Novaspec II spectrophotometer (Biochrom Ltd., Cambridge, UK).

### Skin histology

The effects of dermal patches and sc insulin daily treatments of diabetic rats for 5 weeks on skin morphology were evaluated by histological analysis. The skin tissue samples were fixed in 10% formalin solution, rehydrated in decreasing grades of ethanol and embedded in paraffin wax. These samples (3–5 µm thick) were sectioned with a microm rotary microtome (Robert-Bosch-Straβe, Walldorf, Baden-Württemberg, Germany). Subsequently, the sections were stained with haematoxylin and eosin (H and E), dehydrated in increasing grades of ethanol and cleared in xylene. The processed sections were viewed and captured using a Leica light microscope (Leica Biosystems Peterborough Limited, Peterborough, Berkshire, U.K.).

### Skin permeation studies

To establish whether insulin was transported across skin of STZ-induced diabetic rats following topical application of pectin insulin-containing dermal matrix patches, we monitored the density of phosphorylated insulin receptor substrates (IRS) in skin tissues by immunohistochemical staining. Rats sham treated with drug free pectin hydrogel matrix patches and insulin (175 µg/kg, sc) served as control animals and positive control animals, respectively. Skin samples were also harvested from non-diabetic control animals. Formalin-fixed and paraffin wax embedded skin tissues were sectioned as described in the preceding section and fixed onto pre-cleaned X-tra adhesive slides (Leica Biosystems Peterborough Limited, Peterborough, Berkshire, U.K.). The slides were dewaxed, rehydrated following a standard immunohistochemical protocol and washed twice with Tris-buffered saline with 0.1% Tween 20 (TTBS) (20 mM Tris, 150 mM NaCl, KCl, 0.05% Tween-20) at 2 min interval. The sections were then blocked in 2% BSA for 30 min and the excess buffer was removed with fibre-free filter paper. Subsequently, the sections were incubated in primary antibody (mouse anti-insulin receptor, 1∶500, Abcam, Cambridge, United Kingdom) diluted in 1% BSA for 30 min at room temperature. Thereafter, they were washed thrice as before with TTBS and incubated in peroxidase buffer (Sigma-Aldrich, St. Louis, Missouri, USA) for 10 min. The specimens were then washed as before and incubated in secondary antibody (Rabbit anti-mouse IgG 1∶100, Bio-Rad, Johannesburg, South Africa) for 20 min. The specimens were stained with diaminobenzidine (DAB, Bio-Rad, Johannesburg, South Africa) for 5 min in the dark and then drop-washed in tap water. Finally the slides were counter-stained with Gill’s Haematoxylin (Sigma-Aldrich, St. Louis, Missouri, USA) for 3–5 min and blued in tap water for 5 min. The sections were then dehydrated with increasing degrees of alcohol and cleared with xylene. The coverslips were mounted with permount and the images were captured using Leica scanner SCN 400 (Leica Microsystem CMS, GmbH, Ernst-Leitz-Strasse, Wetzlar, Germany).

### Glycogen synthase and GLUT4 measurements

To further elucidate the effects of insulin-containing dermal patches on diabetic symptoms, the expressions of GLUT4 and glycogen synthase (GS) in liver and gastrocnemius muscle tissues, respectively harvested after 5 weeks of treatment were analyzed using western blotting. Tissue samples (0.1 g) were homogenized on ice in isolation buffer (0.5 mM Na_2_EDTA, 0.1 M KH_2_PO_4_, 0.1 mM dithiothreitol, 0.25 M sucrose) and then centrifuged at 400×g for 10 min (4°C). The protein content was quantified using the Lowry [31] method and all the samples were standardized to one concentration (1 mg/mL). The proteins were then denatured by boiling in laemmli sample buffer (0.5 M Tris-HCl, glycerol, 10% sodium dodecyl sulfate (SDS), 2-mercaptoethanol, 1% bromophenol blue) for 5 min. The denatured proteins (25 µL) were loaded on prepared resolving (10%) and stacking (4%) polyacrylamide gels along with molecular weight marker (5 µL). The gel was electrophoresed for 1 h at 150 V in electrode (running) buffer (Trisbase, glycine, SDS), pH 8.3). Following electrophoresis, the resolved proteins were electro-transferred to an equilibrated polyvinylidene difluoride (PVDF) membrane for 1 h in transfer buffer (192 mM glycine, 25 mM Tris, 10% methanol). After transfer, the membrane was blocked with 5% non-fat dry milk in Tris-buffered saline with 0.1% Tween 20 (TTBS) (20 mM Tris, 150 mM NaCl, KCl, 0.05% Tween-20). The membrane was then immuno-probed with antibodies-GS and GLUT4 (1∶1000 in 1% BSA, Neogen, USA) for 1 h at room temperature (RT). The PVDF membrane was then subjected to 5 washes (10 min each with gentle agitation) in TTBS. Following which, the membrane was incubated in horse radish peroxidase (HRP)-conjugated secondary antibody (rabbit anti-mouse 1∶10000; Bio-Rad) for 1 h at room temperature. After further washing, antigen-antibody complexes were detected by chemiluminescence using the Immune-star™ HRP substrate kit (Bio-Rad, Johannesburg, South Africa). Chemiluminescent signals were detected with the Chemi-doc XRS gel documentation system and analysed using the quantity one software (Bio-Rad, Johannesburg, South Africa). Band intensity analysis was conducted on the resultant bands.

### Statistical analysis

All data were expressed as means ± standard error of means (S.E.M.). Statistical comparison of the differences between the control means and experimental groups was performed with GraphPad InStat Software (version 5.00, GraphPad Software, San Diego, California, USA), using one-way analysis of variance (ANOVA), followed by Tukey-Kramer multiple comparison test. A value of p<0.05 was considered significant.

## Results

### Insulin-loading efficiency

The loading efficiency of different insulin concentrations in PI matrix patches of different insulin concentrations sustain ranged from 76% to 94% (Table 1). The recovery percentages of insulin with the original insulin activity after 2 months storage (75–80%) compared to the initial concentration indicating stability of the patch.

**Table 1:** Insulin-loading in pectin hydrogel matrices and mean loading-efficiencies: Each value represents the mean value of six different samples.

Theoretical insulin inpetr dish (µg)	Actual insulin inpetri dish (µg)	Actual insulinin patch (µg)	Dosageµg/kg	% insulinincorporation	Time inmonths
11.72	11.01±0.97	0.74±0.05	2.47	94	0
23.43	17.81±0.07	1.20±0.01	3.99	76	0
46.86	42.64±0.88	2.87±0.25	9.57	91	0
93.70	74.98±0.58	5.04±0.01	16.80	80	0
	70.28±0.26	4.72±0.09	15.73	75	1
	71.21±0.04	4.79±0.10	15.97	76	2

### Effects of PI patch on the skin

H and E skin stained sections of untreated non-diabetic control, untreated STZ-induced diabetic rats and diabetic animals topically applied insulin-containing dermal patches observed under light microscope showed no significant histological differences in dermis (Fig. 1). Compared to control animals, neither inflammation nor necrosis were detected in the skin as the photomicrographs revealed preserved epidermis and dermis after 5 weeks of daily treatment with insulin-containing dermal patches (Fig. 1). Interestingly, STZ-induced diabetic rats treated with sc insulin injections did not show damage in dermal and epidermal layers of the skin when compared to untreated control animals (Fig. 1).

**Figure 1:** H & E stains illustrating the effects of insulin-containing dermal patches on the morphology of the skin in STZ-induced diabetic rats. Picture A represents intact secretory ducts (white arrow), stratum basale (yellow arrow) and intact sebaceous glands (red arrow) of the untreated control animals. (Mag 8×500 µm). Picture B represents intact secretory ducts (white arrow), uninjured stratum basale (yellow arrow) and intact sebaceous glands (red arrow) of the PI treated animals. (Mag 8×500 µm). Pictures C represents intact secretory ducts (white arrow), uninjured stratum basale (yellow arrow) and intact sebaceous glands (red arrow) of the subcutaneously insulin treated animals (Mag 12×500 µm).

### PI effects on IRS

Skin fragments obtained from STZ-induced diabetic rats for immunohistochemical analysis of IR contained cellular elements from the epidermis and dermis, including hair follicles and glandular structures (Fig. 2). The method control skin section showed faint negative immune-reactivity (Fig. 2A). Untreated non-diabetic rat skin section exhibited intense widespread localization of IRS (Fig. 2B) compared to faint staining of untreated STZ-induced diabetic rats (Fig. 2C). Immunohistochemical staining for phosphorylated IRS in the skin of animals following application of insulin-containing dermal patches and sc insulin treatment for 5 weeks clearly demonstrated widespread localization of IRS in cell bodies of the dermis, collagen and subcutaneous layer (Fig. 2D and Fig. 2E.). The higher magnification of transdermal insulin treated rat skin section confirmed widespread localization of IRS (Fig. 2F).

**Figure 2:** Immunohistochemical micrographs illustrating the effects of transdermally delivered insulin on the expression of Insulin receptor (IR) in skin sections of STZ-induced diabetic rats. The presence of IRS is depicted as brown staining and a method control (A) reveals no immune-reactivity and intense haematoxylin staining (blue) across epidermis and dermis. Untreated non-diabetic rat skin section (B) revealed widespread localization of IRS across the epidermis and dermis. Untreated diabetic control rat skin section (C) exhibited very low immuno-reactivity predominantly in the dermis. Intense immuno-reactivity was observed in the epidemis, dermis and subcutaneous layer of transdermal insulin treated rat skin section (D). Subcutaneous insulin treated rat skin section (E) also exhibited widespread localization of IRS in the epidermis and dermal structures (Mag. 4×500×µm). All the dermal structures including, collagen and hair follicles were positive for IRS with more intensity in the transdermal treatment (F; Mag 27×100 µm).

In summary the widespread localization of IRS in cell bodies of the dermis, collagen and subcutaneous layer evoked by PI-containing dermal patches suggests that the pectin hydrogel insulin patch has the potential to deliver insulin across the skin and into the blood stream.

### OGT responses

OGT responses tests show that blood glucose concentrations were significantly higher in untreated STZ-induced rats at all time-points during the study and the area under the curve (AUC) also increased significantly compared to that in non-diabetic control rats (Fig. 3). Application of insulin-containing dermal patches significantly reduced blood glucose levels in proportion to the concentration of insulin in the hydrogel patches although statistical differences between the doses were not achieved (Fig. 3). In addition, the blood glucose AUC was smaller in treated animals compared with respective control diabetic rats. The administration of insulin (sc) not only demonstrated blood glucose-lowering effects in STZ-induced diabetic rats, but also reduced the AUC. The AUC increases of glucose over baseline values were calculated during OGT responses by the incremental method.

**Figure 3:** Comparisons of OGT responses (A) and AUC_glucose_ (B) of STZ-induced diabetic rats to PI matrix patches of different insulin concentrations with control animals. Values are presented as means, and vertical bars indicate SEM of means (n = 6 in each group). ★p<0.05 by comparison with control animals.

### Insulin pharmacokinetics

Plasma insulin concentrations of untreated STZ-induced diabetic rats were significantly low (p<0.05) in comparison with control non-diabetic animals (Fig. 4). Acute (6 h) and short-term (5 weeks) daily application of PI matrix dermal patches to STZ-induced diabetic rats significantly (p<0.05) elevated plasma insulin concentrations by comparison with untreated diabetic animals. However, the plasma insulin concentrations in animals treated with the high insulin doses (9.57, 16.80 µg/kg) were significantly higher (p<0.05) than those found in diabetic groups treated with low insulin doses (2.47 and 3.99 µg/kg). Interestingly, the plasma insulin concentrations of animals administered sc insulin for 5 weeks were lower compared with those administered insulin through transdermal patches (Fig. 4). These data indicate that insulin was transported from insulin-containing dermal patches into the blood in a dose-dependent manner, with patches containing more insulin leading to a higher insulin concentration in the blood.

**Figure 4:** Comparison of plasma insulin concentrations of STZ-induced diabetic rats to PI matrix patches of different insulin concentrations with control animals. Values are presented as means, and vertical bars indicate SEM of means (n = 6 in each group). ♦p<0.05 by comparison Non-diabetic control. ★p<0.05 by comparison to STZ-induced diabetic control. •p<0.05 by comparison to the lowest dose. ∞ p<0.05 by comparison to transdermally PI treated animals.

### Weight, food and water intake

Table 2 compares the effects of insulin-containing dermal patches on physical parameters of STZ- induced diabetic animals with untreated diabetic and control non-diabetic rats over a period of 5-weeks. Untreated diabetic rats exhibited characteristic signs of diabetes of severe wasting and increased intake of water. There was no change in food intake amongst the groups because all animals were given a standard amount of food (30 g/day) hence no polyphagia was observed. Treatment with PI hydrogel matrix patches containing low doses of insulin (3.99 and 9.57 µg/kg) significantly reduced the weight loss and water intake from week 3 whilst effects of PI patches containing 16.80 µg/kg as well as insulin (175 µg/kg, sc) were observed from week 1.

**Table 2:** Comparisons of the effects of PI matrix patches of different insulin concentrations on body weight, food and water intake in STZ-induced diabetic rats with untreated diabetic rats and control non-diabetic (ND) animals.

		Time (Weeks)				
Parameter	Experimental protocol	1	2	3	4	5
**Food intake (g/100** **g)**	ND control	10±1	9±1	10±1	10±1	11±1
	STZ-control	12±1	13±1	13±1	13±2	14±1
	3.99	11±1	12±1	11±2	11±1	11±1
	9.57	12±1	11±1	11±1	11±1	12±1
	16.80	11±1	11±1	11±1	11±1	11±1
	Sc ins	12±1	11±2	11±1	11±1	11±1
**Water intake (ml/100** **g)**	ND control	20±1	21±2	19±1	20±1	18±1
	STZ-control	58±1*	59±1*	62±1*	63±1*	64±2*
	3.99	56±1*	56±1*	40±2* ^♦^	28±1^♦^	22±1^♦^
	9.57	59±1*	54±2*	48±1* ^♦^	29±1^♦^	20±1^♦^
	16.80	53±1*	50±1*	46±2* ^♦^	26±2^♦^	24±1^♦^
	Sc ins	54±1*	48±1*	38±1* ^♦^	27±1^♦^	18±1^♦^
**% b.wt changes**	ND control	7±1	6±1	8±1	13±2	22±1
	STZ-control	−9±1*	−6±2*	−9±1*	−4±2*	−3±1*
	3.99	−5±1*	−3±1*	2±1^♦^	4±1^♦^	3±1* ^♦^
	9.57	−3±1*	−2±1*	4±1^♦^	3±1^♦^	2±1* ^♦^
	16.80	3±1^♦^	4±1^♦^	4±1^♦^	3±1^♦^	4±2* ^♦^
	Sc ins	6±1^♦^	3±1^♦^	4±2^♦^	2±1^♦^	3±1* ^♦^

Insulin was administered thrice daily for 5-weeks via subcutaneous injection or PI insulin matrices. Data are expressed as mean ± SEM, n = 6 in each group.

*p<0.05 by comparison with control non-diabetic (ND) animals.

♦p<0.05 by comparison with comparison with control STZ-induced diabetic rats.

### Metabolic parameters

Consistent with our use of a diabetic animal model, untreated STZ-induced diabetic rats maintained high blood glucose values throughout the experiment and exhibited extensive depletion of glycogen in liver and muscle tissues by the end of the 5-week study period (Fig. 5 and Table 3). The reduction in glycogen concentration was associated with decreased expressions of the insulin-stimulated GS and GLUT4 in hepatic and skeletal muscle tissues, respectively (Fig. 6). Treatment with PI matrix patch (16.80 µg/kg) as well as insulin (175 µg/kg, sc) restored the expressions of GLUT4 and GS to levels comparable to values of non-diabetic control animals (Fig. 6). The results indicate the potential of insulin medicated adhesive pectin hydrogel skin patch to sustain prolonged controlled insulin release into the bloodstream of STZ-induced diabetic rat with concomitant alleviation of some diabetic symptoms.

**Figure 5:** Comparison of the effects on blood glucose of STZ-induced diabetic rats treated with transdermal PI hydrogel matrix patches on the skin and diabetic rats treated with sc insulin with untreated animals. Animals treated with drug-free pectin and subcutaneous insulin (175 µg/kg) acted as negative and positive controls, respectively. Values are presented as means, and vertical bars indicate SEM of means (n = 6 in each group). ★p<0.05 by comparison with control animals.

**Figure 6:** Comparison of the effects of topically applied PI hydrogel matrix patch and sc insulin on the the insulin-stimulated glycogen synthase (GS) and facilitative glucose transporter (GLUT4) in hepatic and skeletal muscle tissues of STZ-induced diabetic rats, respectively with untreated non-diabetic as determined by Western blotting. Values are expressed as mean ± S.E.M. Values were obtained from Western blots for six preparations. ★p<0.05 by comparison with non-diabetic animals. •p<0.05 by comparison with respective control animals.

**Table 3:** Comparison of hepatic and muscle glycogen concentrations of STZ-induced diabetic rats treated with amidated PI hydrogel patches applied onto the skin with control animals.

	Glucose mmol/L	Glycogen	µg/100 g/tissue
		Hepatic	Skeletal muscle
Non-diabetic control	4.51±0.01	28.42±0.41	2.62±0.32
STZ-control	29.83±2.01^♦^	12.36±0.72^♦^	1.02±0.21^♦^
STZ-TD 3.99	7.13±0.28*	20.08±0.56*	2.02±0.09*
STZ-TD 9.57	6.65±0.18*	21.26±0.64*	2.34±0.20*
STZ-TD 16.80	6.63±0.07*	22.02±1.33*	2.52±0.38*
STZ-SC Ins	5.95±0.11*	21.28±0.94*	2.36±0.21*

Values are presented as means, and vertical bars indicate SEM of means (n = 6 in each group).

*p<0.05 by comparison with respective control animals.

♦p<0.05 by comparison with respective non-diabetic animals.

## Discussion

The current study investigated whether transdermal application of pectin hydrogel insulin matrix patches of different insulin concentrations sustain controlled release of insulin into the bloodstream of streptozotocin (STZ)-induced diabetic rats and alleviate a variety of diabetic symptoms. The results show that topical application of pectin insulin-containing dermal patches to STZ-induced diabetic rats increases plasma insulin concentration, reduces blood glucose and increases liver and muscle glycogen levels as well as the expression of GS and GLUT4 in hepatic and skeletal muscle tissues, respectively. The findings are of considerable importance because application of insulin-containing dermal patches would not only free diabetic patients from some daily bolus injections needed to maintain a constant insulin concentration, but also provide pain-free self-administration of insulin for patients and probably improve compliance. STZ at dose used (60 mg/kg) selective­ly destroys or impairs secretion of insulin from β cells of the pancreas and the systemic changes which occur following this are related to the induced diabetic state [32]–[35]. Indeed, untreated STZ-diabetic rats exhibited significantly low plasma insulin concentration and increased plasma glucose concentrations compared to non-diabetic rats perhaps due to destruction of pancreatic β-cells [32], [33], [36], [37]. PI hydrogel matrix patches evoked changes in blood glucose and plasma insulin concentrations comparable to positive control experiments using sc insulin. The doses of insulin in pectin dermal patches (3.99, 9.57, 16.80 µg/kg) compare with those previously used in human studies (6·25–17·86 µg/kg) [38], [39]. Successful transdermal delivery of insulin was also corroborated with the observation of extensive expression of insulin receptor substrates (IRS) in the skin of STZ-induced rats following application of insulin-containing dermal patches. The insulin receptor (IR), a transmembrane glycoprotein present in virtually all vertebrate tissues undergoes tyrosyl autophosphorylation in response to insulin binding to the extracellular a-subunit [40]–[42]. Conceivably, insulin released from insulin-containing dermal patches enhanced the tyrosine kinase activity of the receptor towards the expression of IRS in the skin of STZ-induced rats [43]–[46] and in insulin target tissues such as skeletal muscle and the liver [43]. The key to strict glycaemic control with exogenous insulin lies with delivery methods that maintain physiological insulin concentrations. Therefore, the pectin insulin-containing dermal patches delivered physiologically relevant amounts of pharmacologically active insulin. A PI hydrogel matrix patch formulation will be easy to use and will not require elaborative devices to prevent drug leakage as in solution formulations. Pectin has been used as a carrier of a wide variety of biologically active agents, for sustained release applications and targeting drugs to the colon for either local treatment or systemic action [14], [34].

The invasive PI dermal patches may offer minimally invasive insulin delivery in clinical applications to perhaps improve insulin bioavailability and patient compliance. Interestingly, comparisons of the effects of pectin hydrogel insulin (PI) matrix patches of different insulin concentrations on plasma insulin concentration and blood glucose lowering could not be separated statistically. The failure to observe these effects cannot be explained by the present study, but may be attributed to the narrow range of the doses used in the present study. Further studies with a wider range of insulin doses are expected to provide this information. Such data would lead to the development of insulin-containing dermal patches into unit dosage forms.

Previously, we reported depletion of glycogen concentration in the liver and skeletal muscle of STZ-induced diabetic rats [47], [48]. Glycogen synthesis in skeletal tissues is dependent on insulin that stimulates translocation of the GLUT4 to the cell membrane to mediate glucose uptake[49]. As assessed by western blotting, PI treatment significantly increased the expression of GS and GLUT4 in the skeletal muscle of STZ-induced diabetic rats suggesting that insulin-containing dermal patches not only improve glycaemic control of STZ-induced diabetic rats, but also increase glucose utilization and transport in hepatic and skeletal muscle tissues, respectively. Decreased glucose transport activity and decreased levels of GLUT4 have been reported in muscle of diabetic patients [50], [51].

We have previously reported that insulin-loaded amidated pectin hydrogel bead formulation sustains controlled insulin release in diabetic rats and lower blood glucose concentration [14]. Building off these previous observations we have further developed an insulin containing cocktail capable of delivering insulin via dermal patches into the bloodstream. The pectin hydrogel matrix cocktail comprised of (a) low methoxy (LM) pectin gelled with calcium ions (b) insulin (c) a transdermal transfer enhancing agent and (d) an antioxidant. The patch concoction did not show any detrimental effects on the morphology of underlying tissues of the skin as evidenced from histological observations. This could be attributed to the protective effect of the antioxidants, vitamin E and eucalyptus oil in the patch. The recovery percentages of insulin with the original insulin activity after 2 months storage proved good stability of the pectin insulin hydrogel insulin matrix patch. The stability of insulin in formulations is an important issue since aggregation of insulin is known to lead to severely reduced biological activity [52].

## Conclusions

The studies reported herein indicate the potential of insulin-containing dermal patch formulation to offer slow controlled release of insulin and alleviate a variety of diabetic symptoms. The limitations of the study include the absence of lipid profile and liver function assessment. In this regard, it is envisaged to utilize the obese Zucker diabetic rat model in future studies.
